# miR-34a Modulates Angiotensin II-Induced Myocardial Hypertrophy by Direct Inhibition of ATG9A Expression and Autophagic Activity

This article has been retracted.

**DOI:** 10.1371/journal.pone.0094382

**Published:** 2014-04-11

**Authors:** Jionghua Huang, Wen Sun, He Huang, Jing Ye, Wei Pan, Yun Zhong, Chuanfang Cheng, Xiangyu You, Benrong Liu, Longgen Xiong, Shiming Liu

**Affiliations:** Department of Cardiology, The Second Affiliated Hospital of Guangzhou Medical University, Guangzhou Institute of Cardiovascular Disease, Guangzhou, China; University of Kansas Medical Center, United States of America

## Abstract

Cardiac hypertrophy is characterized by thickening myocardium and decreasing in heart chamber volume in response to mechanical or pathological stress, but the underlying molecular mechanisms remain to be defined. This study investigated altered miRNA expression and autophagic activity in pathogenesis of cardiac hypertrophy. A rat model of myocardial hypertrophy was used and confirmed by heart morphology, induction of cardiomyocyte autophagy, altered expression of autophagy-related ATG9A, LC3 II/I and p62 proteins, and decrease in miR-34a expression. The in vitro data showed that in hypertrophic cardiomyocytes induced by Ang II, miR-34a expression was downregulated, whereas ATG9A expression was up-regulated. Moreover, miR-34a was able to bind to ATG9A 3′-UTR, but not to the mutated 3′-UTR and inhibited ATG9A protein expression and autophagic activity. The latter was evaluated by autophagy-related LC3 II/I and p62 levels, TEM, and flow cytometry in rat cardiomyocytes. In addition, ATG9A expression induced either by treatment of rat cardiomyocytes with Ang II or ATG9A cDNA transfection upregulated autophagic activity and cardiomyocyte hypertrophy in both morphology and expression of hypertrophy-related genes (i.e., ANP and β-MHC), whereas knockdown of ATG9A expression downregulated autophagic activity and cardiomyocyte hypertrophy. However, miR-34a antagonized Ang II-stimulated myocardial hypertrophy, whereas inhibition of miR-34a expression aggravated Ang II-stimulated myocardial hypertrophy (such as cardiomyocyte hypertrophy-related ANP and β-MHC expression and cardiomyocyte morphology). This study indicates that miR-34a plays a role in regulation of Ang II-induced cardiomyocyte hypertrophy by inhibition of ATG9A expression and autophagic activity.

## Introduction

Cardiac hypertrophy refers to a thickening myocardium, resulting in a decrease in size of the heart chamber. A common cause of cardiac hypertrophy is hypertension or heart valve stenosis. At the cell level, cardiac hypertrophy is generally characterized by an increase in the size of cardiomyocytes, without increase in cell numbers, and by cytoskeletal reorganization. At the molecular level, cardiac hypertrophy shows an increased expression of fetal-type genes [1], [2]. Physiologically, cardiac hypertrophy is initially an adaptive response to stress overload. However, the continued presence of hypertrophic growth often carries a poor prognosis that may result in heart failure and sudden death of patients [3], [4].

To date, appropriate therapy and prevention methods of cardiac hypertrophy progression have had limited success because the pathophysiological mechanisms responsible for cardiac hypertrophy development remain to be defined. To this end, a previous study showed that cardiac hypertrophy induced by pressure-overload stress triggers cardiomyocyte autophagy [5]. Moreover, cardiomyocyte excessive autophagy may lead to cardiomyocyte death [6] although physiological levels of autophagy are essential in eukaryotic cells to eliminate damaged proteins and organelles as part of the maintenance of cell homeostasis. This excessive or deficient autophagy may therefore contribute to disease pathogenesis. As the only integral membrane ATG protein, ATG9A is localized in the phagophore/pre-autophagosomal structure (PAS) [7], [8] and is an essential protein in the autophagic process.

In addition, microRNAs (miRNAs) are a class of endogenous non-coding RNAs and modulate gene expression at the post-transcriptional level by binding to the seed-matched sequence of the 3′-UTR region in their target mRNAs, which results in either degradation or translational repression of target gene expression. Altered expression of miRNAs has been associated with development of cardiac hypertrophy [9]. Recent studies have further indicated that miRNAs also plays a role in cardiac development and physiology [10]. For example, miR-34a is a multifunctional regulator, which is involved in cell division [11], senescence [12], apoptosis [13] and proliferation [14] through regulating the expression of its target genes. Using microarray profiling, Cheng at al. [15] demonstrated that miR-34a was aberrantly expressed in hypertrophic mouse hearts. However, the molecular mechanism regulating cardiac hypertrophy by miR-34a has been poorly understood. Yang et al. [16] elucidated that miR-34a modulated Caenorhabditis elegans lifespan via the repression of ATG9A-mediated autophagic activities. Angiotensin II (Ang II) is a critical growth factor and mediates cardiac hypertrophy, and its receptors can regulate cardiomyocyte autophagy [17].

However, it is unknown whether and how these factors work together to regulate cardiac hypertrophy, whether ATG9A mediated autophagic activity is excessively activated in Ang II induced cardiomyocyte hypertrophy, and whether miR-34a can modulate Ang II-induced cardiomyocyte hypertrophy by targeting ATG9A expression. Thus, we hypothesized that during development of cardiac hypertrophy, miR-34a could modulate Ang II induced myocardial hypertrophy by repression of ATG9A mediated autophagic activity. We took this novel approach to help better understand the molecular mechanisms of cardiac hypertrophy development in order to develop a prospective therapeutic target for control of cardiac hypertrophy in the future.

## Materials and Methods

### A rat animal model of cardiac hypertrophy

In this study, we performed an animal experiment to produce cardiac hypertrophy in rat. Specifically, male Sprague-Dawley rats from the Guangdong Medical Laboratory Animal Centre (Guangzhou, China) were randomly divided into 2 groups, i.e., Sham group (n = 6) and transverse abdominal aortic constriction (TAAC) group (n = 8) as described [18]. This animal model produced a well-established rat cardiac hypertrophy by transverse abdominal aortic banding. The TAAC group of rats was anaesthetized with ketamine (80 mg/kg, IP) and xylazine (5 mg/kg, IP) under sterile conditions and the abdominal aorta was ligated between the abdominal aorta and anterior mesenteric artery with a blunted 5-gauge needle (external diameter = 0.5 mm) and a 4-0 nylon suture. After that, the needle was quickly removed. However, in the Sham group, rats only underwent exposure of the aorta.

### Evaluation of cardiac hypertrophy in vivo

Cardiac hypertrophy of this animal model was evaluated by echocardiography, histopathological analysis of heart size, the ratio of heart weight to body weight (HWI), and cardiomyocyte size in hematoxylin and eosin (H&E)-stained heart cross-sections [19]–[21]. In brief, 4 weeks after the surgery, we evaluated the left ventricular wall thickness and ejection fraction, heart chamber size using transthoracic echocardiography (Philips IE33, Netherlands) with a 7.5 MHz sector scan probe after 4 weeks under mild pentobarbital anesthesia (15 mg/kg, IP). The left ventricular end-diastolic and end-systolic dimension (LVIDd and LVIDs), left ventricular posterior wall end-diastolic and end-systolic thickness (LVPWd and LVPWs), left ventricular ejection fraction (EF%) were measured from M-mode traces. Following completion of the transthoracic echocardiography, rats were sacrificed with an overdose of pentobarbital. The hearts were then carefully removed from the rats for HW measure HWI calculation. The hearts were fixed in 4% paraformaldehyde, dehydrated, and embedded in paraffin. Tissue sections were prepared by leveling the papillary muscle and measuring the cardiomyocyte size after H&E staining. The images of tissue sections were acquired using a fluorescence microscope (Nikon, Eclipse, Ti-U), and morphometric analysis was performed (software used was NIS-Elements F 4.0).

### Construction of plasmid vectors carrying ATG9A CDS and 3′-UTR

pRC/CMV_2_ over-expression vector and pGL3 luciferase reporter vector were purchased from Invitrogen (Carlsbad, CA) and Promega (Madison, WI), respectively. Coding sequence (CDS) fragments of ATG9A were PCR-amplified from rat cDNA with two linkers (i.e., Hind III and Xba I) and then inserted into pRC/CMV_2_ using T4 DNA ligase. Having been confirmed by DNA-sequencing, this plasmid was named as pRC/CMV_2_-ATG9A and used in vitro to produce expression of ATG9A protein. Furthermore, rat genomic DNA containing the 3′-untranslated region (3′-UTR) of ATG9A was extracted from rat blood using an E.Z.N.A™ Blood DNA Kit (Omega, Norcross, USA) according to the manufacturer's instructions. After which the ATG9A 3′-UTR and a mutation sequence were amplified from rat genomic DNA using a fusion PCR and inserted into the ECOR I and Xba I sites of a pGL3 luciferase reporter vector. Following confirmation by DNA-sequence, these plasmids were named as pGL3-ATG9A 3′-UTR-Wild Type and pGL3-ATG9A 3′-UTR-Mutant. The pRL-TK (Promega) was used as an endogenous control.

### Cell culture and treatment

Rat ventricular cardiomyocytes were isolated by enzymatic digestion from 1- to 3-day-old neonatal Sprague-Dawley rats and cultured as described previously [22]. The following treatments were pursued for the cell cultures, i.e., stimulation of cardiomyocytes with 1 µmol/L Ang II (human angiotensin II from Sigma, St Louis, MO); Lentivirus carrying miR-34a mimics (miR-34a), miR-34a inhibitor (miR-34a inhibitors), negative control of miR-34a, ATG9A siRNA, or negative control-siRNA, all having been purchased from the corporation of GenePharma, China (sequences are shown in Table 1). For lentiviral transductions, 4×10^5^ of cardiomyocytes were transduced with 20 µl lentivirus (10^9^ TU/ml) and polybrene (at a final concentration of 5 µg/ml). pRC/CMV_2_-ATG9A and vector control were transfected with Lipofectamine LTX and PLUS Reagents (Invitrogen) according to the manufacturer's instructions.

**Table 1:** PCR primer and siRNA sequences.

Gene name	RT-PCR primer
U6	5′-CGCTTCACGAATTTGCGTGTCAT-3′
miR-34a	5′-GTCGTATCCAGTGCGTGTCGTGGAGTCGGCAATTGCACTGGATACGACACAACCAG-3′

Gene name	q-PCR primer
U6	5′-CGCTTCACGAATTTGCGTGTCAT-3′
	5′-GCTTCGGCAGCACATATACTAAAAT-3′
miR-34a	5′-GCCCTGGCAGTGTCTTAG-3′
	5′-CAGTGCGTGTCGTGGAGT-3′
18s	5′-ACCGCAGCTAGGAATAATGGA-3′
	5′-GCCTCAGTTCCGAAAACCA-3′
ANP	5′-GGGGGTAGGATTGACAGGAT-3′
	5′-CTCCAGGAGGGTATTCACCA-3′
β-MHC	5′-CCTCGCAATATCAAGGGAAA-3′
	5′-TACAGGTGCATCAGCTCCAG-3′
ATG9A	5′-AAAGCCTGGTGCTGTCTGAATA-3′
	5′-CTCTCTCCACTCTCATCACTCTCC-3′

Gene name	siRNA sequences
Negative control for ATG9A siRNA	5′-GTTCTCCGAACGTCACGTCAAGAGATTACGTGACACGTTCGGAGAATT-3′
ATG9A siRNA	5′-GGTTCACATGTATGCTCATTGTTCAAGAGACAATGAGCATACATGTGAACCTT-3′
Negative control for miR-34a	5′-TTCTCCGAACGTGTCACGTTTC-3′
miR-34a mimics	5′-TGGCAGTGTCTTAGCTGGTTGT-3′
miR-34a inhibitors	5′-ACAACCAGCTAAGACACTGCCA-3′

### Dual luciferase reporter assay

To assess whether miR-34a regulates ATG9A expression, we performed a dual luciferase reporter assay. In brief, neonatal rat cardiomyocytes were seeded for 5×10^4^ cell per well into 24 well plates. After 5 days culture, the cells were transduced with a lentivirus containing miR-34a mimic, miR-34a inhibitor or miR-34a negative control and 12 hours later, pGL3 luciferase reporter vector including 3′-UTR of ATG9A (with the wild type or mutant type) was cotransfected with the pRL-TK vector into the cardiomyocytes using Lipofectamine LTX and PLUS Reagents (Invitrogen) for 48 hours. After that, the cardiomyocytes were collected and lysized to measure the luciferase activities of Firefly and Renilla using a Lumat LB 9507 (Berthold technologies, Bad Wildbad, Germany). The pRL-TK vector provided constitutive Renilla luciferase expression and was used as an internal control to normalize the Firefly luciferase activity.

### RNA isolation and quantitative real-time polymerase chain reaction (qRT-PCR)

Total cellular RNA was isolated from tissues or cultured cells using Trizol (Invitrogen) and cDNA was synthesized using a PrimeScript II 1st Strand cDNA Synthesis kit (TakaRa, Japan) according to the manufacturers' protocols. qRT-PCR was then performed using the SYBR Premix Ex Taq™ II Kit (TakaRa) in a LightCycler480 SW 1.51 System from LightCycler480 II (Roche, Basel, Switzerland). U6 small nuclear RNA and 18S mRNA were used as the internal controls for miRNA and mRNA detection, respectively. The relative expression levels of miRNA and mRNA were calculated using the 2^−ΔΔCT^ method. The primer sequences are shown in Table 1.

### Protein extraction and Western blot

Total cellular protein was isolated from cardiac tissue and cardiomyocytes using a NP-40 lysis buffer (Beyotime, Shanghai, China). The protein concentrations were then assessed by a Bradford assay (Bio-Rad, Hercules, CA). After that, equal amounts of protein samples (40 µg) were separated by sodium dodecyl sulfate-polyacrylamide gel electrophoresis (SDS-PAGE) and transferred onto a polyvinylidene fluoride (PVDF) membrane. For Western blotting, the PVDF membrane was blocked with 5% skimmed milk powder for 1 hour and then incubated with a rabbit monoclonal antibody against ATG9A (Epitomics, Burlingame, CA), a rabbit monoclonal antibody against GAPDH (Epitomics, Burlingame), a rabbit monoclonal antibody against p62 (Abcam, Cambridge, UK), or a polyclonal antibody against LC3 (Cell Signaling Technology, Danvers, MA) at 4°C overnight. On the next day, the membranes were washed with phosphate buffered saline-Tween 20 (PBS-T) thrice and then further incubated with an anti-rabbit peroxidase-conjugated secondary antibody (BOIWORLD, Wuhan, China). The immunological complexes were then visualized by chemiluminescence BeyoECL Plus (Beyotime). Protein expression was normalized to levels of GAPDH expression.

### Transmission electron microscopy

The tissue and cell samples were processed as described previously [23] and the transmission electron microscopy was performed using a Tacnai 12 Spirit Twin transmission electron microscope at a magnification of ×13500. For each tissue or cell section, 10 images were taken randomly from different fields to calculate the number of autophagic vacuoles, with the investigator blinded as to the origin of each image. The morphological criteria [24] of autophagosomes or autolysosomes were set as follows: at the ultrastructural level, a double-membrane structure containing undigested cytoplasmic contents, which had not fused with lysosomes, or intracellular organelles such as mitochondria, and fragments of the endoplasmic reticulum (ER).

### Flow cytometric detection of autophagic vacuoles

Neonatal rat cardiomyocytes were inoculated into 6-well plates and treated with different procedures for 72 hours. After which the cells were collected and washed with PBS for flow cytometric analysis using a BD Cytofix/Cytoperm™ Fixation/Permeabilization Kit (BD Biosciences, San Diego) according to the manufacturer's protocol. Briefly, the cells were fixed and lysized with BD fixation/permeabilization, and washed by BD Perm/wash™ Buffer. The anti-LC3 antibody (Cell Signaling Technology) and goat anti-rabbit IgG-affinity pure, FITC conjugate secondary antibody (ImmunoReagents, Raleigh, NC) were diluted with BD Perm/wash™ buffer. The cells were first incubated with an anti-LC3 antibody and then a goat anti-rabbit IgG secondary antibody in 4°C for 30 minutes each. LC3 protein served as a marker for autophagic vacuoles and labeled by fluorescent secondary antibody. The ratio of autophagic vacuoles was detected using BD Accuri C6 Flow Cytometer and analyzed with BD accuri C6 software.

### Confocal microscopy

The cells were harvested and fixed with 3.7% formaldehyde at 37°C and permeabilized with 1% Trion X in PBS-T for 15 minutes. Next, the cells were incubated with Alexa Fluor555 Phalloidin (1∶35, Invitrogen) for 25 minutes and then stained with the chromatin dye, DAPI (300 nmol/L from Invitrogen) for 5 minutes. Finally, cell images were acquired using a Zeiss LSM 710 confocal microscope (Carl Zeiss, Germany). For each sample, 5 images from different fields were randomly selected and used to measure the average cell area (the cardiac muscle fiber surface area) using Image-Pro Plus 6.0 software.

### Statistical analysis

The experimental data were expressed as mean ± SEM. The Shapiro-Wilk test was used to assess whether the data followed a normal distribution. For two group comparisons, a Student's t test was performed, while for more than two group comparisons, an ANOVA was used. All tests were two-sided and a significance level of a P value less than 0.05 was defined as statistical significant (SPSS 18.0 software, SPSS, Chicago, IL).

### Ethics statement

All animal protocols were approved by the review board of the Animal Care and Ethics Committee of Guangzhou Medical University.

## Results

### An animal model of myocardial hypertrophy, dysregulation of miR-34a expression, and autophagic activity

In this study, we first produced a rat model of cardiac hypertrophy through transverse abdominal aortic banding. The results of transthoracic echocardiography showed in Table 2, compared with the Sham group, the cardiac LVPW, IVS, and LVIDs of rats in the TAAC group were markedly increased. The HWI was greater in the TAAC group of rats than in those of the Sham group. The whole heart sections, cut at the papillary muscle level, showed that the heart volume was significantly expanded, while the papillary muscles and trabeculae carneae cordis were much coarser in appearance in the TAAC group than in the Sham group (Fig. 1A). H&E stained tissue sections from the TAAC group displayed a lightly stained color in the regions of myocardial hypertrophy with inhomogeneous staining and numerous nuclear-free regions with an increased nucleolar density in regions of muscle fiber atrophy. In addition, the related area of the cardiomyocytes was markedly enlarged in rats that had undergone the TAAC operation (Fig. 1B). All the results elucidated that a cardiac hypertrophy model in rats had been successfully established.

**Figure 1:** A rat model of cardiac hypertrophy assessed by histopathology. (**A**) Representative images of rat transthoracic echocardiography in Sham operation and transverse abdominal constriction (TAAC) after 4 weeks of animal experiments. H&E staining of heart tissue sections from Sham operation and transverse abdominal constriction (TAAC) after 4 weeks of animal experiments and images were acquired by scanning. The graph shows the heart and body weight and the heart weight index (HWI), which was calculated by heart weight to body weight ratio. *P<0.05 compared to the Sham rats. (**B**) H&E staining of heart tissue sections from Sham and TAAC rats and images were taken with scanning, the scar bar: 50 µm. Regions of myocardial hypertrophy were lighter in color with homogeneous staining, and showed numerous nuclear-free regions, with an increased nucleolar density in regions of muscle fiber atrophy. The graph summarizes data on relative cell area that were determined from local cardiac HE-stained paraffin sections and presented as mean ± SEM. *P<0.05 compared to the Sham rats.

**Table 2:** Cardiac structure and systolic function.

	Sham (n = 6)	TAAC (n = 8)
IVSd (10^−3^ cm)	127.83±4.71	196.25±9.53 *
IVSs (10^−3^ cm)	216.5±16.43	320.13±15.32 *
LVIDd (10^−3^ cm)	577.33±22.05	537.13±15.37
LVIDs (10^−3^ cm)	358.17±19.24	263.88±9.62 *
LVPWd (10^−3^ cm)	153.17±8.16	217.38±12.72 *
LVPWs (10^−3^ cm)	217.33±0.79	321.25±8.24 *
EF (%)	85.7±1.69	88.38±0.92

Data were expressed as mean ± SEM, *P<0.05 compared to the Sham rats.

Next, we assessed autophagy and expression of autophagy-related protein LC3 II/I and p62, the two established markers for autophagic activity, in these rat heart tissues. The data showed that the number of autophagic vacuoles was induced in the TAAC group of rats when compared to the Sham rats (Fig. 2A) and that expression of autophagy-related gene, ATG9A and LC3 II/I was also induced in TAAC rats, but expression of p62 protein (an adaptor protein involved in linking polyubiquitylated protein aggregates and the autophagic machinery) was repressed in TAAC (Fig. 2B). Since miR-34a was aberrantly expressed in hypertrophic mouse heart [15], we thus assessed miR-34a expression in these rat heart tissues and found that miR-34a expression was significantly downregulated in the TAAC group of rats compared to that of the Sham group (Fig. 2C). These data suggest autophagy and expression of these genes may participate in development of cardiac hypertrophy.

**Figure 2:** Altered miR-34a and ATG9A expression, autophagic vacuoles, and autophagy in a rat cardiac hypertrophy model. (**A**) The autophagic vacuoles in left ventricular tissues from Sham and TAAC rats were analyzed 4 weeks after surgery by transmission electron microscopy (arrows indicated). Magnification, ×13500. Scale bar: 1 µm. The graph summarizes the data on changed autophagic vacuoles in TAAC vs. Sham rats. *P<0.05 compared with the Sham group. (**B**) Gene expression analyzed by qRT-PCR and Western blotting. The graph quantifies the Western Blot data. *P<0.05 compared with the Sham group. (**C**) qRT-PCR detection of miR-34a expression. U6 was used as an internal control. Data are presented as means ± SEM. *P<0.05 compared with the Sham group.

### Ang II-induced myocardial hypertrophy and ATG9A and miR-34a expression in vitro

As a critical growth factor, Angiotensin II can mediate cardiac hypertrophy; thus, we used it to establish an in vitro cardiomyocytes hypertrophic model in this study. The cardiomyocytes were treated with 1 µmol/L Ang II and then evaluated morphologically and through the expression of hypertrophy-related genes. Compared to the control cardiomyocytes, Ang II-treated cardiomyocytes showed markedly increased expression of hypertrophy-related genes and cell area (Fig. 3A). Moreover, expression of ATG9A mRNA and protein was also upregulated (Figs. 3C and D). In contrast, miR-34a expression was downregulated (Fig. 3B). These results elucidate to the fact that both ATG9A and miR-34a are involved in development of myocardial hypertrophy induced by Ang II.

**Figure 3:** Altered miR-34a and ATG9A expression in Ang II-induced myocardial hypertrophy model in vitro. (**A**) Evaluation of Ang II-induced myocardial hypertrophy in terms of hypertrophy-related gene expression (ANP and β-MHC) and morphological changes. Morphological changes were measured by confocal microscopy after staining with Alexa Fluor555 Phalloidin and DIPI. The graph summarized the data on changed hypertrophy-related gene expression and cell morphology. *P<0.05 compared with controls (Con). (**B**) qRT-PCR detection of miR-34a. U6 was used as an internal control. Data are presented as means ± SEM. *P<0.05 compared with Con. (**C**) qRT-PCR analysis of ATG9A expression. 18s was used to normalize ATG9A expression. Data are presented as means ± SEM. *P<0.05 compared with Con. (**D**) ATG9A protein expression was analyzed by Western blotting. The graph quantified Western Blot data. *P<0.05 compared with Con.

### Effect of miR-34a on direct suppression of ATG9A expression in cardiomyocytes

To demonstrate the role of miR-34a in the regulation of ATG9A expression, we performed the luciferase assay to directly assess whether miR-34a can bind to the 3′-UTR of ATG9A mRNA (Fig. 4A) using a bioinformatics approach (www. target scan.org). As shown in Fig. 4B, after cardiomyocytes were transfected with pGL-3-ATG9A 3′-UTR-Wild Type, transduction with miR-34a mimics resulted in a 45% reduction in the relative luciferase activity, compared to cells treated with a negative control. In contrast, transduction with miR-34a inhibitor resulted in a 1.38-fold increase in the relative luciferase activity, compared to cells treated with a negative control. However, after in cardiomyocytes were transfected with pGL-3-ATG9A 3′-UTR-Mutant Type, the effects of miR-34a was lost (Fig. 4B).

**Figure 4:** miR-34a regulation of ATG9A expression. (**A**) Sequence alignment between miR-34a and the 3′-UTR of ATG9A in different species and schematic diagram of construction of pGL3-ATG9A 3′-UTR-Wild Type and pGL3-ATG9A 3′-UTR-Mutant Type plasmids. (**B**) Luciferase assay. The report plasmid in which the luciferase coding sequence was fused to ATG9A-3′-UTR-Wild or ATG9A-3′-UTR-Mutant and miR-34a mimics, miR-34a inhibitors, and negative control were cotransfected into cardiomyocytes. Renilla luciferase activity was normalized to firefly luciferase activity. *P<0.05 compared with NC group. (**C**) qRT-PCR in detection ATG9A mRNA level after transfection of miR-34a mimics or inhibitor into cardiomyocytes. Expression values were normalized to the 18S housekeeping gene. *P<0.05 compared with NC group. (**D**) Western blot analysis of ATG9A protein after transfection of miR-34a mimics or inhibitors into cardiomyocytes. *P<0.05 compared with NC group.

Meanwhile, we determined the effect of miR-34a on regulation of ATG9A expression. The data showed that compared to the negative control, miR-34a was unable to significantly express ATG9A mRNA as shown by real-time PCR analysis (Fig. 4C). But transduction of miR-34a mimics reduced expression of ATG9A protein by a 38% decrease, while transduction of miR-34a inhibitors induced levels of ATG9A protein by 1.7-fold (Fig. 4D), suggesting that miR-34a suppressed expression of ATG9A protein at the post-transcriptional level.

### Effect of ATG9A expression on regulation of autophagic activity in cardiomyocytes

We then further confirmed whether ATG9A expression alters autophagic activity by performing several interventional experiments. First, we induced ATG9A expression in cardiomyocytes with Ang II or transfection of pRC/CMV_2_-ATG9A and found that, compared to the control, either Ang II or transfection of pRC/CMV_2_-ATG9A were able to induce ATG9A expression (Figs. 3C, D and 5A, C) and in turn altered autophagic activity (Figs. 5C and 6A). In contrast, Ang II could induce ATG9A expression and autophagic activity, but knockdown ATG9A expression using ATG9A siRNA antagonized Ang II induced effect in cardiomyocytes (Figs. 5B, D and 6B). TEM data also showed similar results (Fig. 6D). Taken together, these data demonstrated that the alteration in cardiomyocyte autophagy was cause by ATG9A expression in Ang II-stimulated cardiomyocytes.

**Figure 5:** Effect of ATG9A expression on regulation of autophagy-activated marker protein levels in cardiomyocytes. (**A**) qRT-PCR. The cardiomyocytes were transfected with ATG9A cDNA or vector control and then subjected to qRT-PCR analysis of AGT9A mRNA. *P<0.05 compared with vector Control. (**B**) qRT-PCR. The cardiomyocytes were treated with negative control lentivirus or Ang II plus ATG9A siRNA or plus negative control lentivirus and then subjected to qRT-PCR analysis of AGT9A mRNA. *P<0.05 compared with negative Control; ^#^P<0.05 compared with Ang II + NC. (**C**) Western blot. The cardiomyocytes were treated with 1 µmol/L Ang II or control (Con) or transfected with ATG9A cDNA or vector control and then subjected to Western blot. *P<0.05 compared with Control. (**D**) Western blot. The cardiomyocytes were treated with negative control lentivirus or Ang II plus ATG9A siRNA or plus negative control lentivirus and then subjected to Western blot. *P<0.05 compared with negative Control; ^#^P<0.05 compared with Ang II + NC. The graphs are quantified data from the Western blots.

**Figure 6:** Effects of ATG9A and miR-34a expression on Ang II-induced autophagic activity in cardiomyocytes. (**A**) Flow cytometry. The autophagic vacuoles were detected by using flow cytometry with an anti-autophagy marker protein (LC3) in the cardiomyocytes. The graph summarizes the data of flow cytometry. *P<0.05 compared with Control group. (**B**) Flow cytometry. The graph summarizes data from the flow cytometry. *P<0.05 compared with NC group, ^#^P<0.05 compared to Ang II + NC. (**C**) Flow cytometry. The graph summarizes data from the flow cytometry. *P<0.05 compared with NC group, ^#^P<0.05 compared to Ang II + NC. (**D**) TEM. The autophagic vacuoles were detected and calculated by transmission electron microscopy (as indicated by the arrows). Magnification of images: ×13500. The graph is the quantitative data from the transmission electron microscopy. Data are presented as means ± SEM *P<0.05 compared with Control group; ^#^P<0.05 compared to Ang II + NC. (**E**) TEM. Magnification of images: ×13500 and ×46000, respectively. The graph is the quantitative data from the transmission electron microscopy. Data are presented as means ± SEM *P<0.05 compared with NC group; ^#^P<0.05 compared to Ang II + NC.

### Effect of miR-34a on suppression of autophagic activity in Ang II-treated cardiomyocytes

We then assessed the effect of miR-34a on suppression of autophagic activity in Ang II-treated cardiomyocytes. Autophagic activity can be measured using flow cytometry and TEM. Compared to the negative control, Ang II treatment increased the ratio of autophagic activity in cardiomyocytes, whereas overexpression of miR-34a using miR-34a mimics decreased the ratio of autophagic activity induced by Ang II (Fig. 6C). Moreover, TEM data confirmed the effects of miR-34a in suppression of autophagic activity induced by Ang II (Fig. 6E).

### Effect of ATG9A expression on induction of cardiomyocyte hypertrophy

Next, we assessed the effect of ATG9A expression on the induction of cardiomyocyte hypertrophy. Cardiomyocyte hypertrophy was detected using two hypertrophic gene markers ANP and β-MHC in cardiomyocytes. Both Ang II treatment and transfection of ATG9A cDNA induced ATG9A expression in cardiomyocytes and upregulated levels of ANP and β-MHC mRNA, whereas the negative control or Ang II treatment plus ATG9A siRNA infection reduced the levels of ANP and β-MHC mRNA in cardiomyocytes compared to Ang II treatment plus the negative control (Figs. 3A and 7A). Moreover, we also measured cell area (size) as further evidence of hypertrophy and found similar data as the expression of ANP and β-MHC mRNA (Figs. 3A and 7B). The data demonstrated that Ang II-induced cardiomyocyte hypertrophy was through upregulation of ATG9A expression in cardiomyocytes.

**Figure 7:** Effect of altered ATG9A expression on Ang II-induced myocardial hypertrophy. (**A**) qRT-PCR. The cardiomyocytes transfected with ATG9A cDNA or vector control or lentiviral control or treated with Ang II plus ATG9A siRNA or lentiviral control and then subjected to qRT-PCR analysis of the hypertrophy-related genes ANP and β-MHC mRNA. (**B**) Confocal microscopy. The cardiomyocyte morphology was measured by a confocal microscope after staining with Alexa Fluor555 Phalloidin and DIPI. The graph summarizes the confocal microscopy data. *P<0.05 compared to control; ^#^P<0.05 compared to Ang II + NC.

### Effect of miR-34a expression on regulation of Ang II-induced cardiomyocyte hypertrophy

We then determined whether miR-34a expression can modulate Ang II-induced cardiomyocyte hypertrophy in vitro. Our data showed that 1 µmol/L Ang II-treated cardiomyocytes induced cardiomyocyte hypertrophy in terms of expression of the cardiomyocyte hypertrophy markers ANP and β-MHC mRNA and a cell area of cardiomyocytes, and decreased miR-34a expression (Figs. 3A and B). However, in Ang II-induced hypertrophic cardiomyocytes, upregulation of miR-34a by miR-34a mimics antagonized Ang II-stimulated cardiomyocyte hypertrophy, whereas knockdown of miR-34a by miR-34a inhibitors aggravated Ang II-induced cardiomyocyte hypertrophy (Figs. 8A and B). These data further indicate that miR-34a plays an important role in regulation of Ang II-induced cardiomyocyte hypertrophy through inhibition of ATG9A expression.

**Figure 8:** Effects of miR-34a on regulation of Ang II-induced myocardial hypertrophy. (**A**) qRT-PCR. The cardiomyocytes were treated with control lentivirus or Ang II plus control lentivirus or Ang II plus miR-34a mimics or Ang II plus miR-34a inhibitors and then subjected to qRT-PCR analysis of the hypertrophy-related genes ANP and β-MHC mRNA. *P<0.05 compared to NC; ^#^P<0.05 compared to Ang II + NC. (**B**) Confocal microscopy. The cardiomyocyte morphology was measured by Confocal microscopy after staining with Alexa Fluor555 Phalloidin and DIPI. The graph summarizes the confocal microscopy data. *P<0.05 compared to NC; ^#^P<0.05 compared to Ang II + NC.

## Discussion

In this study, we first produced a rat model of myocardial hypertrophy using the TAAC operation and then an in vitro cardiomyocytes hypertrophic model using Ang II treatment, ATG9A cDNA transfection, or lentiviral infection of miR-34a inhibitor, or miR-34a mimics, or ATG9A siRNA. We found that the rat myocardial hypertrophy heart tissues increased autophagic activity and upregulated expression of autophagy-related ATG9A and LC3 II/I proteins, but reduced p62 and miR-34a expression. Inhibition of p62 vs. induction of LC3 II/I expression further confirmed increased autophagy activity in this animal model. Furthermore, our in vitro data showed that Ang II-induced cardiomyocyte hypertrophy had decreased expression levels of miR-34a, but ATG9A expression was elevated. However, lentiviral transduction of miR-34a expression modulates Ang II-induced cardiomyocyte hypertrophy and expression of hypertrophy-related genes (i.e., ANP and β-MHC). We then further confirmed that miR-34a was able to directly bind to ATG9A 3′-UTR and suppressed the levels of ATG9A protein, whereas upregulation of ATG9A expression increased autophagic activity, cardiomyocytes area and expression of hypertrophy-related genes, but miR-34a activity was antagonized by Ang II treatment. Our data demonstrated that miR-34a did play an important role in regulation of Ang II-induced cardiomyocyte hypertrophy by inhibition of ATG9A expression and autophagy. Future studies will verify miR-34a as a target for clinical control of myocardial hypertrophy.

Indeed, level of miR-34a expression is various in different pathological conditions; for example, in the ageing heart [25] or myocardial infarction [26], miR-34a was up-regulated, whereas in a number of cancers, such as lung cancer and bladder cancer [27], [28], miR-34a expression was markedly down-regulated. Moreover, level of miR-34a expression might not be the same in different pathological stages of cardiac remodeling due to pressure overload via transverse aortic constriction [15], [26]. In hypertrophic stage of myocardial remodeling, miR-34a expression was down-regulated [15], but it was up-regulated in the myocardial remodeling of heart failure stage [26]. Actually, in our current data on miR-34a expression were consistent with a previous microarray profiling study [15]. However, the molecular mechanism regulating cardiac hypertrophy by miR-34a has been poorly understood. Our current study revealed the underlying molecular events, which further supports this previous study [15]. However, further studies are needed to clarify the importance of the role which miR-34a plays in cardiomyocyte hypertrophy because other studies have revealed the role of different miRNAs in cardiomyocyte hypertrophy. For example, previous published studies showed that inhibition of miR-1 [29], miR-23a [30], or miR-133 [31] expression accelerated cardiaomyocyte hypertrophy, while other studies demonstrated that myocardial hypertrophy was regulated by miR-22 and miR-30a in vivo and in vitro [32], [33]. Similarly, transient gain- and loss-function of miR-26a in cardiomyocytes also confirmed that cardiomyocyte hypertrophy was modulated by miR-26a expression [34]. These data indicate that a number of miRNAs function in the regulation of cardiomyocyte hypertrophy. As we known, each miRNA, such as miR-34a, can target multiple genes. For example, a previous study demonstrated that an ectopic expression of miR-34a substantially inhibited growth of IMR90 cells and molecularly, miR-34a suppressed expression of c-MET and cell cycle-related genes [13]. Another study confirmed these data in esophageal cancer cells whereby transfection of miR-34a into various esophageal cancer cell lines suppressed tumor cell growth and expression of c-MET and cyclinD1 [35]. In addition, miR-34a is a downstream gene of the tumor suppressor p53 protein [13], [36]. In our current study, we demonstrated the role of miR-34a in the suppression of cardiomyocyte hypertrophy by directly targeting ATG9A expression. Indeed, previous studies demonstrated that ATG9A plays an important role in cardiomyocyte autophagy and cardiac hypertrophy [37], [38]. However, further studies will be needed to verify our current data on miR-34a controlled ATG9A-induced cardiac hypertrophy.

Furthermore, at the physiological level the role of autophagy is to maintain normal cell and tissue homeostasis by elimination of damaged proteins and organelles in the cells. However, excessive or deficient autophagy could contribute to disease pathogenesis. In the stage of myocardial hypertrophy induced by pressure overload, Zhu et al [5] and Nakai et al [6] elucidated that myocardial autophagy was excessively activated. Other recent studies further confirmed that autophagy activation was a key participant in pressure-overload induced myocardial hypertrophy [39], [40]. But in pressure overload-induced heart failure, myocardial autophagy was impaired [41]. While cardiac remodeling was in myocardial hypertrophy stage, excessive autophagy may be a protective reaction. Conversely, when it came into heart failure stage, the myocardial autophagy ability was markedly impaired and contributed to the progression of disease. Molecularly, both LC3 and p62 are markers of measuring the autophagy activity, but their expression is in opposite direction, i.e., increased autophagy activity showed upregualtion of LC3 expression but downregulation of p62 expression [42], [43]. Indeed, our current study showed increased autophagy activity and upregualtion of LC3 expression, but downregulation of p62 expression in the rat model of cardiomyocyte hypertrophy and after miR-34a expression.

Recent studies on miRNAs regulation of cardiac autophagy showed that miR-204 [44] and miR-30a [33] could modulate myocardial autophagy via targeting LC3-II or Beclin-1, respectively. Moreover, miR-212 and miR-132 [45] were able to regulate autophagy in cardiomyocytes via their commonly targeting gene of Foxo3 expression. Many previous studies have reported that miR-34a is not only involved in regulation of the cell cycle, differentiation, and apoptosis through expression of the target genes, such as CDC25C, CREP and Bcl-2 [12]–[14], but is also implicated in the regulation of autophagic activity [46], [47]. Thus, miR-34a may have various roles in different types of cells during various physiological and pathological conditions. In our current study, neonatal cardiomyocytes stimulated by Ang II were transduced with miR-34a mimics and it was shown that miR-34a was able to inhibit autophagic activity, and that these cells when transduced with miR-34a inhibitor caused enhancement of autophagic activity. Molecularly, expression of ATG9A protein was altered by Ang II and miR-34a mimics. This protein not only is a transmembrane protein and localized at both pre-autopahgosomal structure (PAS) and multiple peripheral structures, but is also one of the characterized 31 Atg proteins to participate in autophagic activation [38], [39]. Our current study demonstrated that ATG9A can be directly targeted by miR-34a, which further confirmed a previous study [16] using Hela and HEK293 cells. Thus, our current finding indicated that miR-34a can suppress expression of ATG9A, thereby suppressing the autophagic activity in cardiomyocytes.

In summary, the present study shows that miR-34a can modulate Ang II-induced cardiomyocyte hypertrophy. This effect of regulation is implemented by direct inhibition of ATG9A expression and autophagic activity. Our studying provides a valuable clue for developing a prospective therapeutic target for control of cardiac hypertrophy in the future.
